# Mulberry Leaf Flavonoids Inhibit Liver Inflammation in Type 2 Diabetes Rats by Regulating TLR4/MyD88/NF-*κ*B Signaling Pathway

**DOI:** 10.1155/2022/3354062

**Published:** 2022-07-06

**Authors:** Yuhui Duan, Hongyu Dai, Yongcheng An, Long Cheng, Lu Shi, Yinglan Lv, Huimin Li, Chen Wang, Changhao He, Huilin Zhang, Yan Huang, Wanxin Fu, Yanyan Meng, Baosheng Zhao

**Affiliations:** ^1^Department of Pharmacology, School of Chinese Materia Medica, Beijing University of Chinese Medicine, Beijing 102488, China; ^2^College of Life Sciences, Beijing University of Chinese Medicine, Beijing 102488, China; ^3^Beijing Research Institute of Chinese Medicine, Beijing University of Chinese Medicine, Beijing 100029, China

## Abstract

The incidence of liver-related complications in type 2 diabetes mellitus (T2DM) is rapidly increasing, which affects the physical and mental health of T2DM patients. Mulberry leaf flavonoids (MLF) were confirmed to have certain effects on lowering blood glucose and anti-inflammation. In this study, the high-fat diet (HFD) + STZ method was used to establish T2DM rat model and the MLF was administered by gavage for eight weeks. During the experiment, body weight and blood glucose level were measured at different time points. The pathological changes of rat liver were observed by H&E staining. The serum glucolipid metabolic indicators of serum, fasting insulin (FINS), and inflammatory factors levels were detected by ELISA. The expression levels of toll-like receptor 4 (TLR4), TNF receptor-associated factor 6 (TRAF6), myeloid differentiation factor 88 (MyD88), inhibitor of NF-*κ*B alpha (I*κΒα*), p-I*κΒα*, and nuclear factor kappa-B (NF-*κ*B)/p65 protein in liver tissue were measured by Western Blot. After 8 weeks' MLF treatment, the blood glucose of rats showed a downward trend; glycolipid metabolism level and insulin resistance were improved, which suggested that MLF could improve the disorder of glucose and lipid metabolism. The pathological damage and inflammation of the liver in T2DM rats were significantly improved, the levels of related serum inflammatory factors were reduced, and the expression of liver tissue-related proteins was downregulated. Our results indicated that MLF could reduce blood glucose and inhibit the development of liver inflammation. The mechanisms may be associated with the activation of TLR4/MyD88/NF-*κ*B signal pathway to reduce the levels of inflammatory factors in serum.

## 1. Introduction

Diabetes is the third major disease that seriously threatens human health at present. Because of its high morbidity, mortality, and disability rate and multicomplications, it seriously threatens patients' lives and brings heavy psychological and economic burdens to families and society [1]. According to the ninth edition of diabetes map of the International Diabetes Federation in 2019, there are about 463 million diabetes patients in the world at present, and it is estimated that the number will reach 700 million by 2045 [2]. The main types of diabetes are type 1 diabetes mellitus (T1DM), type 2 diabetes mellitus (T2DM), and gestational diabetes mellitus (GDM). Among them, T2DM accounts for over 90% of the total number of diabetes mellitus [3]. T2DM is a common chronic metabolic disease, and it is generally believed that its pathogenesis is related to decreased islet function and insulin resistance (IR) [4]. However, because of its diverse etiology and complex pathogenesis, there is no radical cure drug at present. Therefore, it is crucial to study the mechanism of T2DM and its complications to find new therapeutic approaches for T2DM.

The liver is one of the main organs for controlling metabolic homeostasis; it is also a major target tissue for insulin to exert its effect, which is involved in maintaining the balance of blood glucose, as well as an effective organ for inflammatory mediators [5]. T2DM is apt to cause hepatic diseases, such as nonalcoholic fatty liver, liver inflammation, liver fibrosis, and so on [6]. More than 50% of diabetic patients suffer from liver diseases, and 60–70% of T2DM obese patients are prone to liver steatosis. However, researchers pay little attention to diabetic liver injury, especially inflammatory lesions [7]. Toll-like receptor (TLRs) is a kind of pattern recognition receptors, and TLR4 is an important member of TLRs family, which mediates the inflammatory response of the body [8]. When the body is damaged, TLR4 is activated. TLR4 is transmitted through MyD88-dependent pathway, which promotes the binding of phosphorylated IL-1 receptor associated kinase (IRAK) to TRAF6 and activates inhibitor of nuclear factor kappa-b kinase (IKK), thus activating NF-*κ*B [9]. Activated NF-*κ*B can promote the release of TNF-*α*, IL-1*β*, and IL-6. The study has confirmed that mulberry leaves can inhibit the production of NF-*κ*B by regulating TLR4 signaling pathway, thus inhibiting the release of inflammatory factors [10].

Flavonoids are one of the natural active components in mulberry (*Morus alba* L.) leaves, accounting for 1% ∼ 3% of the dry weight of mulberry leaves [11]. Studies have shown that total flavonoids of mulberry leaves have pharmacological effects, such as antioxidant, hypoglycemic, hypolipidemic, and antitumor [12]. Our previous study found that the hypoglycemic effect of mulberry leaf is related to the inhibition of *α*-glucosidase [13], the immune inflammation induced by TLRs signaling pathway, the regulation of insulin signaling pathway [14], and the regulation of brown fat metabolism [15]. However, more early researches paid more attention to the total mulberry leaf extract, and less research focused on the total flavonoids in mulberry leaves and the impact on the liver inflammation. To further enrich the pharmacological effects of total flavonoids from mulberry leaves, this study observed the effects of total flavonoids from mulberry leaves on blood glucose and liver inflammation in T2DM rats and preliminarily explored its anti-inflammatory mechanism based on TLR4-MyD88-NF-*κ*B signaling pathway.

## 2. Materials and Methods

### 2.1. Preparation of Total MLF

The dried mulberry leaves were purchased from Beijing Bencao Fangyuan Pharmaceutical Group Co., Ltd. (20200630). Mulberry leaves were crushed by a pulverizer, sieved with 40 mesh sieve, and ultrasonically treated with 80% ethanol (output power 500 W, temperature 50°C, and ratio of material to liquid 1 : 25 g/ml) for 75 min. Anhydrous ethanol was added at a ratio of 1 : 8 g/mL, and precipitating with ethanol was carried out for 2 times, 12 hours each time. The supernatant was purified by AB-8 macroporous resin. The eluate was evaporated with a rotary evaporator until no ethanol smell was found, and freeze-drying method was used to obtain mulberry leaf total flavonoids. By the quantitative determination of our research group, the average content of mulberry leaf was 58.29%. UHPLC-Q Exactive MS technology results confirmed that various flavonoid components such as rutin, isoquercetin, and astragalin were present in the MLF of this experiment. The HPLC results confirmed that the contents of flavonoids rutin, isoquercetin, and astragalin in the extract (MLF) were 5.26 mg/g, 4.82 mg/g, and 2.63 mg/g.

### 2.2. Animals and Treatments

Forty male SPF SD rats, with weight of 180g∼200 g, were purchased from Beijing Sibeifu Biotechnology Co., Ltd., and the experimental animal production license number was SYXK (Jing) 2019-0010. The rats were raised in a specific pathogen-free animal laboratory affiliated to the Experimental Animal Center of Beijing University of Chinese Medicine, License no. SCXK (Jing) 2016-0038. The animal protocol in this study was reviewed and approved by the medical and experimental animal ethics committee of Beijing University of Chinese Medicine (no. BUCM-4-2020091504–3153).

After one week's adaptive feeding, 6 rats were randomly selected as normal groups according to their body weight and fed with normal maintenance feed. The rest of the rats were given high-sugar and high-fat diet for 4 weeks, then fasted for 12 hours, and intraperitoneally injected with 1% STZ sodium citrate buffer at 35 mg/kg, while the normal group was intraperitoneally injected with 1% sodium citrate buffer. After 72 hours, blood was collected from tail vein to measure their fasting blood glucose. Taking blood glucose ≥ 11.1 mmol/L as the modeling standard, 4 unqualified rats were excluded. The model rats were randomly divided into T2DM group, metformin (200 mg/kg) group, high-dose group of mulberry leaf flavonoids (HMLF, 300 mg/kg), medium-dose group of mulberry leaf flavonoids (MMLF, 150 mg/kg), and low-dose group of mulberry leaf flavonoids (LMLF, 75 mg/kg). MLF was dissolved with 0.5% sodium carboxymethyl cellulose, and rats in each treatment group were given MLF by gavage. The administration volume is 1 mL/100 g body weight. Rats in other groups were given the same amount of sodium carboxymethyl cellulose once a day for 8 weeks.

### 2.3. Glucose Tolerance Tests

The fasting weight and blood glucose of rats in each group were measured every week. One week before the end of the experiment, after fasting for 12 h, 50% glucose (2 g/kg) was gavaged. The blood glucose at 0, 15, 30, 60, and 120 min was measured, respectively, and the area under the curve (AUC) was calculated based on the blood glucose curve:

AUC (mmol/h·L) = (BG 0 min + BG 15 min) × 1/4 × 1/2 + (BG 15 min + BG 30 min) × 1/4 × 1/2 + (BG 30 min + BG 60 min) × 1/2 × 1/2 + (BG 60 min + BG 120 min) × 1/2 (BG is the blood glucose value at each time point).

### 2.4. Biochemical Analysis

Blood was collected from abdominal aorta of rats, and serum was separated by centrifugation. TC, TG, HDL-C, and LDL-C were measured by biochemical method. Serums IL-1*β*, IL-6, and TNF-*α* were detected by ELISA.

### 2.5. Histological Staining

The rat liver tissue was fixed with 4% paraformaldehyde solution for 24 hours, and dehydration, embedding, slicing, and H&E staining were performed successively. Pathological changes of liver tissue were observed under light microscope.

### 2.6. Western Blot Analysis

The liver was weighed and ground with liquid nitrogen. The milled tissue powder was added into lysis solution containing RIPA (tissue weight: volume of lysis solution 20 mg:150–250 *μ*L) for lysis. BCA protein detection kit was used to detect protein concentration. The total protein (10 *μ*g) of each sample was added to SDS-PAGE gel electrophoresis to separate the protein and transferred to PVDF membrane (Millipore). The PVDF membrane containing protein was incubated in a closed solution for 2 hours and then incubated in the required primary antibody, including TLR4 antibody (1 : 500, ab13556; Abcam), MyD88 antibody (1 : 1000, ab219413; Abcam), TRAF6 (1 : 1000, ab33915; Abcam), I*κ*B antibody (1 : 2000, ab76429; Abcam), P-I*κ*B antibody (1 : 1000, 2859 S; Abcam), NF-*κ*B antibody (1 : 2000, ab16502; Abcam), and *β*-actin antibody (1 : 10000, 20536-1-AP; Proteintech), incubated at 4°C overnight. After incubating with HRP-conjugated AffiniPure Goat Anti-Rabbit IgG (H + L) (1 : 5000, SA00001-2, Proteintech) and HRP-conjugated AffiniPure Goat Anti-Mouse IgG (H + L) (1 : 5000, SA00002-1, Proteintech) for 1 h, the PVDF membrane was washed with solution TBST, treated with chemiluminescence reagent, taken photos by exposure, and performed quantitative analysis with Image-Pro Plus 6.0.

### 2.7. Statistical Analysis

All the data in this study were statistically analyzed by SPSS 25.0 software and were expressed as mean ± SD. The differences between the two groups were analyzed by independent *t*-test, and multiple groups were analyzed by using the one-way analysis of variance (ANOVA) followed by SNK-*q* test. *p* value< 0.05 was considered as statistically significant.

## 3. Results

### 3.1. Effect of MLF on Body Weight and Liver Index of T2DM Rats

Compared with the normal group, the weight of rats in the model control group decreased significantly (*p* < 0.01). Compared with the model group, there was no statistical difference in the weight of rats in each administration group (Figure 1(a)). Compared with the normal group, the liver index in T2DM group was significantly enhanced (*p* < 0.01). Compared with T2DM rats, the liver index of HMLF, MMLF, and LMLF rats decreased significantly (*p* < 0.01) (Figure 1(b)). It is suggested that the total flavonoids of mulberry leaves could reduce the body weight and liver index of T2DM rats.

### 3.2. Effect of MLF on Glucose Metabolism in T2DM Rats

As shown in Figure 2(a), compared with the normal group, the rats in T2DM group were in hyperglycemia state during the experiment (*p* < 0.01). Compared with T2DM group, the fasting blood glucose of rats in metformin group significantly decreased from the 4th week to 8th week (*p* < 0.05 or *p* < 0.01). The fasting blood glucose of rats in HMLF group and MMLF group decreased significantly from the 5th to 8th week (*p* < 0.01). The fasting blood glucose of rats in LMLF group significantly decreased from the 5th to 8th week (*p* < 0.05).

As shown in Figures 2(b) and 2(c), the blood glucose increased obviously after being given 50% glucose and reached the highest value at 30 min in each group and showed a downward trend. Compared with the control group, the AUC of OGTT in T2DM group increased significantly within 0–120 min (*p* < 0.01). Compared with T2DM group, metformin, HMLF, MMLF, and LMLF groups decreased significantly at 0 min (*p* < 0.01), and AUC decreased significantly (*p* < 0.01 or *p* < 0.05). It is suggested that MLF could reduce blood glucose and maintain glucose tolerance in T2DM rats.

### 3.3. Effect of MLF on Insulin

Serum insulin level was measured by enzyme labeling method in rats of each group after 8 weeks of administration. As shown in Figures 3(a) and 3(b), compared with the normal group, the fasting insulin level and HOMA-IR in T2DM group were significantly higher (*p* < 0.01). Compared with T2DM group, fasting insulin level in normal group and each administration group decreased, and HOMA-IR value decreased significantly (*p* < 0.01). It is suggested that total flavonoids of mulberry leaves could improve insulin sensitivity in T2DM rats.

### 3.4. Effect of MLF on Lipid Metabolism

As shown in Figure 4, compared with the normal group, the levels of TC, TG, and LDL-C in T2DM group were significantly increased (*p* < 0.01), while the levels of HDL-C were significantly decreased (*p* < 0.01). Compared with T2DM group, the levels of TC, TG, and LDL-C were significantly decreased (*p* < 0.01) and HDL-C was significantly increased (*p* < 0.01). The results showed that total flavonoids of mulberry leaves could improve the disorder of blood lipid metabolism in T2DM rats.

### 3.5. Effects of MLF on Pathological Sections of Liver

Pathological sections of the liver were stained with H&E staining. As shown in Figure 5, the results showed that no obvious abnormality was found in the overall morphological structure of liver in the control group, each administration group and hepatocytes, and no obvious abnormality was found in the morphological structures of hepatic lobular, central vein, and portal area. Microscopic examination of the liver in the T2DM group revealed vacuolar degeneration, which was characterized by the presence of vacuoles in the hepatocytes, with incomplete fragmentation of the cytoplasm, which were widely distributed in the liver, ranging from mild to severe. There was also lymphocyte infiltration, which was characterized by scattered or small aggregates of lymphocytes, with a small number of neutrophils partially observed.

### 3.6. Effects of MLF on Inflammation Indicators

As shown in Figure 6, compared with the normal group, the levels of IL-6, IL-1*β*, and TNF-*α* in the T2DM group were significantly increased (*p* < 0.01). Compared with the T2DM group, the expression levels of IL-6, IL-1*β*, and TNF-*α* in each administration group were significantly reduced (*p* < 0.01). The results suggested that MLF could reduce the inflammation level of liver in T2DM rats.

### 3.7. Effects of MLF on Protein Expression of TLR4, MyD88, TRAF6, I*κ*B, p-I*κ*B, and NF-*κ*B in Liver

As shown in Figure 7, compared with the normal group, the protein expression levels of TLR4, MyD88, TRAF6, I*κ*B, p-I*κ*B, and NF-*κ*B in the model group were significantly increased (*p* < 0.01). Compared with the T2DM group, the expression levels of TLR4, MyD88, TRAF6, and NF-*κ*B proteins in the HMLF group were significantly downregulated (*p* < 0.01). Meanwhile, after MLF treatment, the ratio of p-I*κ*B/I*κ*B was also significantly reduced (*p* < 0.01). The results confirmed that MLF can inhibit liver inflammation in T2DM rats by regulating the TLR4/MyD88/NF-*κ*B pathway.

## 4. Discussion

T2DM is a common chronic metabolic disease, with various pathogenic factors and complex pathogenesis, which poses a serious threat to human health. Liver lesions are one of the common complications of diabetes. In the state of T2DM, fat accumulates in the liver and gradually forms the liver inflammation [16]. The inflammatory reaction in the liver further accelerates the development of T2DM, and the two diseases promote each other, eventually causing irreversible damage to the body. Flavonoids are one of the main active components of mulberry leaves, mainly including quercetin, rutin, isoquercetin, kaempferol, and astragalin. Studies have confirmed that MLF can scavenge oxygen free radicals, regulate energy homeostasis, repair damaged islet cells, promote insulin secretion, and regulate glucose metabolism [17]. MLF have been demonstrated to effectively reduce blood glucose levels in diabetic mice by regulating intestinal microecological disorders [18]. Rutin could facilitate signal transduction and activated state of insulin IRS-2/PI3K/Akt/GSK-3*β* signal pathway, promote hepatocyte proliferation, reduce blood glucose level and generation of AGEs, and improve liver damage in T2DM mice. In addition, the previous study of our research group found that rutin has potential therapeutic implications for the treatment of obesity and T2DM. Rutin decreased blood glucose in db/db mice, inhibited hepatic lipid accumulation, and improved glucose and lipid metabolism disorders; these pharmacological effects may be related to the promotion of the mRNA expression of the adipocyte thermogenic genes MCT1, MCT1, ACSM3, CPT-1*α*, and CPT-1*β*, activation of BAT and induction of browning of IWAT, and increasing the concentration of SCFA-producing enzymes, promoting the production of SCFA [19]. Isoquercetin has been shown to reduce serum ALT, AST, improve IR, increase HDL-C, reduce degeneration, necrosis, and apoptosis of liver tissue, and prevent liver damage caused by T2DM [20]. Moreover, isoquercetin in MLF has significant antidiabetic effects by increasing glucose uptake and differentiation in HepG2 cells by regulating AGEs/RAGE and p38 MAPK/NF-*κ*B pathways, increasing PPAR*γ*, C/EBP*α*, and SREBP-l expression in 3T3-L1 cells, and inhibiting AGEs-induced damage and apoptosis by glutathione cells [21]. The results of this study have shown that MLF can regulate the inflammatory response in the liver, by improving the glucolipid metabolism disorder in T2DM rats, and provide the experimental basis for the hypoglycemic effect of MLF and the inhibition of inflammatory injury in the liver.

T2DM, characterized by hyperglycemia, is a high-risk metabolic disease involving metabolic disorders, such as systemic glucose and lipid metabolism [22]. In this experiment, the T2DM rat model was replicated by high-fat diet feeding combined with intraperitoneal injection of STZ, and the blood glucose, OGTT, and INS were measured. Blood glucose values reflect the changes of instantaneous blood glucose; OGTT reflects the body's regulation of blood glucose; and FINS and HOMA-IR reflect the ability of insulin to decompose blood glucose [23]. The detection of three indicators together could reflect the changes of blood glucose level of diabetic rats more comprehensively and objectively. The results showed that, compared with the control group, T2DM group showed a significant increase in blood glucose. The intervention of MLF significantly reduced blood glucose, indicating that MLF has a certain hypoglycemic effect. OGTT refers to oral glucose tolerance test, which is used to understand the function of islet *β* cells and the body's ability to regulate blood glucose, and is widely used in the clinical diagnosis of diabetes [24].

OGTT results showed that MLF can regulate blood glucose status and improve abnormal glucose tolerance of the body. FINS and HOMA-IR results showed that the serum INS level in T2DM group was significantly higher than that of control group, while the insulin resistance index was significantly increased. Insulin resistance of T2DM rats was significantly reduced in all administration groups. These three results indicated that MLF can improve the insulin resistance, reduce the level of blood glucose and insulin, and improve glucose metabolism disorder. Lipid metabolism disorders will cause dyslipidemia, *β* -cell insulin secretion function is damaged, and excessive fatty acids hinder the removal of glucose and eventually lead to T2DM [25]. Therefore, improving lipid metabolism is an important means in the treatment of T2DM. In this experiment, TC, TG, LDL, and HDL related indicators of lipid metabolism were detected. The results showed that the related lipid indicators were significantly reduced after administration of MLF, confirming that MLF can improve lipid metabolism. In summary, MLF can improve the glucolipid metabolic disorders, thus affecting the occurrence and development of T2DM.

The liver is an important organ involved in glycolipid metabolism in the body and also the main target organ for insulin resistance [26]. Hepatic insulin resistance increases the free fatty acids, and the fat in the liver accumulates to form fatty liver, which finally leads to inflammation, necrosis, and fibrosis of the fatty liver. At the same time, it will lead to decreased glycogen synthesis and enhanced gluconeogenesis, which will increase blood glucose and lead to the occurrence of T2DM [27]. In this study, we found that the liver index increased significantly in T2DM group, which may be related to the lipid metabolism disorder caused by T2DM leading to the accumulation of liver fat. After MLF administration, the liver index in each group was significantly decreased, and the results confirmed that MLF can reduce IR, thereby affecting liver weight and improving liver lipid metabolism disorder.

Inflammation is an important factor affecting the occurrence and development of T2DM. Inflammation can cause IR and impaired islet *β* cell function. More and more studies have suggested that T2DM is a “chronic low-grade inflammation state” [28]. When IR is in the state, various mediators related to metabolic syndrome in lymphocytes, macrophages, endothelial cells, and adipocytes are activated, and these cells can recognize the corresponding receptors, activate the inflammatory pathway, and release a variety of inflammatory mediators, including TNF-*α*, IL-6, and IL-1*β* [29]. Under hyperglycemia, the production of IL-1*β*, IL-6, and TNF-*α* is promoted, thereby accelerating the apoptosis of islet *β* cells and inducing islet failure [30]. Compared with other tissues, liver itself contains a large number of intrinsic macrophages [31]. When inflammation occurs, the liver is infiltrated by peripheral inflammatory cells, and macrophages are activated, constantly aggravating the development of inflammation [32]. Therefore, in the T2DM state, it will lead to inflammatory damage to the liver. In this experiment, we studied the serum-related inflammatory indicators, such as IL-1*β*, IL-6, and TNF-*α*, and found that compared with the control group, the related inflammatory indicators in the T2DM group were significantly expressed, and the expression level of related inflammatory indicators was significantly reduced after administration of MLF. The experimental results confirmed that MLF effectively improve liver inflammation caused by T2DM.

TLRs are pattern recognition receptors that can detect and respond to specific conservative motifs related to microbial activity, recognize exogenous pathogens, induce the activation of multiple rapid-response genes, and produce multiple effector molecules to participate in the body's defense responses [33]. TLR4 plays a key role in the treatment of diabetes and its complications [34, 35]. TLRs stimulation signals are transmitted to MyD88 through intracellular TIR regions. The linker protein of MyD88 interacts with IRAK to phosphorylate IRAK [36]. Phosphorylated IRAK recruits TRAF6 to react, leading to the activation of NF-*κ*B inhibitory protein (I*κ*K) and phosphorylation of I*κ*B to activate NF-*κ*B, which enters the nucleus [37].

NF-*κ*B is a major transcription factor responsible for the regulation of congenital and adaptive immune responses and a key factor for the initiation of inflammatory response and regulation of gene transcription. NF-*κ*B is involved in the occurrence and development of various diseases, such as immunity and inflammation in the body [38]. NF-*κ*B is a heterodimer that contains two protein subunits, p65 and p50 [39]. Under normal conditions, NF-*κ*B binds to protein I*κ*B in an inactive state. While under pathological conditions, I*κ*B kinase is phosphorylated by NF-*κ*B-induced kinase and transported to the nucleus through a series of pathways, where it initiates gene transcription and releases cytokines [40]. NF-*κ*B has a strong transcriptional regulatory function, which is able to expand the inflammatory process of the disease by activating multiple inflammatory genes. After NF-*κ*B enters the nucleus, it induces the expression of specific genes, synthesizes IL-1*β*, IL-6, TNF-*α*, and other cytokines, and releases them to the outside of the cell to aggravate the inflammatory expression level in the body [41]. The results of this experiment showed that MLF improves the liver inflammatory injury in T2DM rats by inhibiting proteins, such as TLR4, MyD88, TRAF6, I*κ*B*α*, p-I*κ*B*α*, and NF-*κ*B p65.

## 5. Conclusion

Inflammation plays an essential role in the development of T2DM. T2DM aggravates the development of liver inflammation, which itself may also contribute to T2DM. Therefore, how to alleviate liver inflammation in T2DM is particularly important. This study demonstrated that MLF can reduce blood glucose of T2DM, improve glucolipid metabolism disorders, enhance insulin sensitivity, and exert the pharmacodynamic activity of improving T2DM. At the same time, MLF can also reduce the liver index of T2DM rats and inhibit relevant inflammatory indicators, thereby regulating the development of liver inflammation in T2DM rats. These effects may be related to the fact that MLF reduces the levels of related inflammatory factors in the body by regulating the proteins related to TLR4, MyD88, TRAF6, I*κ*B, p-I*κ*B, and NF-*κ*B.

However, this study also has shortcomings. This study mainly discusses the liver inflammatory reaction caused by T2DM and MLF on its treatment, but the liver is an important metabolic organ; fat accumulation accelerated liver inflammatory infiltration. In this study, only the serum lipid metabolism indexes were determined, and the liver lipid metabolism was poorly studied; we will increase the liver lipid metabolism mechanism, further improving the effect of MLF in improving T2DM liver damage. Furthermore, although MLF is already a kind of active ingredient in mulberry leaves, it is unknown which monomer or which monomers play the main hypoglycemic effect. We will carry out further experimental studies on one or more monomers in MLF.

## Figures and Tables

**Figure 1:** (a) Effects of MLF treatment on body weight (g $\bar{x}\pm s$). (b) Effects of MLF treatment on fasting blood glucose (g/g, $\bar{x}\pm s$). Data are presented as mean ± SD. ^#^*p* < 0.05, ^##^*p* < 0.01 versus control group; ^*∗*^*p* < 0.05, ^*∗∗*^*p* < 0.01 versus T2DM group.

**Figure 2:** (a) The effect of MLF on blood glucose in rats (mmol/l, $\bar{x}\pm s$). (b) The effect of MLF on OGTT in rats (mmol/l, $\bar{x}\pm s$). (c) AUC of OGTT value ($\bar{x}\pm s$).

**Figure 3:** (a) Effects of MLF on INS level in rats (mU/L, $\bar{x}\pm s$). (b) Effects of MLF on insulin resistance index of rats ($\bar{x}\pm s$).

**Figure 4:** (a) Effect of MLF on serum TC level in rats (mmol/L, $\bar{x}\pm s$). (b) Effects of MLF on serum TG level in rats (mmol/L, $\bar{x}\pm s$). (c) Effects of MLF on serum HDL-C level in rats (mmol/L, $\bar{x}\pm s$). (d) Effects of MLF on serum LDL-C level in rats (mmol/L, $\bar{x}\pm s$).

**Figure 5:** Effect of MLF on pathological sections of rat liver. (a) Control group. (b) T2DM group. (c) Metformin group. (d) HMLF group. (e) MMLF group. (f) LMLF group.

**Figure 6:** (a) The effect of MLF on serum IL-1*β* level in rats (pg/ml, $\bar{x}\pm s$). (b) The effect of MLF on serum IL-6 level in rats (pg/ml, $\bar{x}\pm s$). (c) The effect of MLF on serum TNF-*α* level in rats (pg/ml, $\bar{x}\pm s$).

**Figure 7:** Effect of MLF on protein expression of TLR4/MyD88/NF-*κ*B signaling pathway.

## Data Availability

The data used to support the findings of this study are available within the article.

## References

[1] Jing Z., Chu J., Imam Syeda Z. (2019). Catastrophic health expenditure among type 2 diabetes mellitus patients: a province-wide study in Shandong, China. *Journal of Diabetes Investigation*.

[2] International Diabetes Federation (2019). *IDF Diabetes Atlas*.

[3] Zheng Y., Ley S. H., Hu F. B. (2018). Global aetiology and epidemiology of type 2 diabetes mellitus and its complications. *Nature Reviews Endocrinology*.

[4] Halim M., Halim A. (2019). The effects of inflammation, aging and oxidative stress on the pathogenesis of diabetes mellitus (type 2 diabetes). *Diabetes & Metabolic Syndrome: Clinical Research Reviews*.

[5] Tanase D. M., Gosav E. M., Costea C. F. (2020). The intricate relationship between type 2 diabetes mellitus (T2DM), insulin resistance (IR), and nonalcoholic fatty liver disease (NAFLD). *Journal of Diabetes Research*.

[6] Xu X. J., Wang W. Q., Lin L., Chen P. (2020). Liraglutide in combination with human umbilical cord mesenchymal stem cell could improve liver lesions by modulating TLR4/NF-kB inflammatory pathway and oxidative stress in T2DM/NAFLD rats. *Tissue and Cell*.

[7] Lyall M. J., Thomson J. P., Cartier J. (2020). Non-alcoholic fatty liver disease (NAFLD) is associated with dynamic changes in DNA hydroxymethylation. *Epigenetics*.

[8] Bielaszewska M., Mellmann A., Karch H., Marejková M., Bauwens A., Kunsmann-Prokscha L. (2018). Enterohemorrhagic *Escherichia coli* O157 outer membrane vesicles induce interleukin 8 production in human intestinal epithelial cells by signaling via Toll-like receptors TLR4 and TLR5 and activation of the nuclear factor NF-*κ*B. *International Journal of Medical Microbiology*.

[9] Justino P. F. C., Franco A. X., Pontier-Bres R. (2020). Modulation of 5-fluorouracil activation of toll-like/MyD88/NF-*κ*B/MAPK pathway by Saccharomyces boulardii CNCM I-745 probiotic. *Cytokine*.

[10] Jeong J. W., Lee H. H., Lee K. W. (2016). Mori folium inhibits interleukin-1*β*-induced expression of matrix metalloproteinases and inflammatory mediators by suppressing the activation of NF-*κ*B and p38 MAPK in SW1353 human chondrocytes. *International Journal of Molecular Medicine*.

[11] Riche D. M., Riche K. D., East H. E., Barrett E. K., May W. L. (2017). Impact of mulberry leaf extract on type 2 diabetes (Mul-DM): a randomized, placebo-controlled pilot study. *Complementary Therapies in Medicine*.

[12] Feng G. Y., Liu Y. Y., Li Y. H., Zhou L. (2020). Hypoglycemic and hypolipidemic effects and mechanisms of flavonoids from mulberry leaves and its application in animal production. *Chinese Journal of Animal Nutrition*.

[13] Tang M. M., Liu Y., Tian S. M. (2015). *α*-glucosidase inhibition by different extracts of folium mori in vitro assay. *Journal of Xinjiang Medical University*.

[14] Tian S. M., Wang M., Liu C. Y., Zhao H. B., Zhao B. S. (2019). Mulberry leaf reduces inflammation and insulin resistance in type 2 diabetic mice by TLRs and insulin Signalling pathway. *BMC Complementary and Alternative Medicine*.

[15] Cheng L., Wang J., An Y. (2021). Mulberry leaf activates brown adipose tissue and induces browning of inguinal white adipose tissue in type 2 diabetic rats through regulating AMPK signaling pathway. *British Journal of Nutrition*.

[16] Wang Y. H., Viscarra J. H., Kim S. J., Sul H. S. (2015). Transcriptional regulation of hepatic lipogenesis. *Nature Reviews Molecular Cell Biology*.

[17] Chen L. L., Liu W., Chen J. G., Bu W. L. (2010). Mechanism of mulberry leaf flavonoids on blood glucose regulation in diabetic mice. *Chinese Journal of Clinical Pharmacology*.

[18] Zhang L. W., Su S. L., Dai X. X. (2019). Regulation of the mulberry leaf effective fraction on the gut microbiota of db/db mice. *Journal of Pharmacy*.

[19] Cheng L., Shi L., He C. H. (2022). Rutin-activated adipose tissue thermogenesis is correlated with increased intestinal short-chain fatty acid levels. *Phytotherapy Research*.

[20] Huang X. L., He Y., Ji L. L. (2017). Hepatoprotective potential of isoquercitrin against type 2 diabetes-induced hepatic injury in rats. *Oncotarget*.

[21] Li J. S., Ji T., Su S. L. (2022). Mulberry leaves ameliorate diabetes via regulating metabolic profiling and AGEs/RAGE and p38 MAPK/NF-*κ*B pathway. *Journal of Ethnopharmacology*.

[22] Hansel B., Giral P., Gambotti L. (2017). A fully automated web-based program improves lifestyle habits and HbA1c in patients with type 2 diabetes and abdominal obesity: randomized trial of patient E-coaching nutritional support (the ANODE study). *Journal of Medical Internet Research*.

[23] Peddinti G., Bergman M., Tuomi T., Groop L. (2019). 1-Hour post-OGTT glucose improves the early prediction of type 2 diabetes by clinical and metabolic markers. *Journal of Clinical Endocrinology and Metabolism*.

[24] Coccia F., Testa M., Guarisco G. (2020). Insulin resistance, but not insulin response, during oral glucose tolerance test (OGTT) is associated to worse histological outcome in obese NAFLD. *Nutrition, Metabolism, and Cardiovascular Diseases*.

[25] Erion D. M., Park H. J., Lee H. Y. (2016). The role of lipids in the pathogenesis and treatment of type 2 diabetes and associated co-morbidities. *BMB Reports*.

[26] Li S., Huang Q., Zhang L. (2019). Effect of CAPE- p NO 2 against type 2 diabetes mellitus via the AMPK/GLUT4/GSK3*β*/PPAR*α* pathway in HFD/STZ-induced diabetic mice. *European Journal of Pharmacology*.

[27] James O. F., Day C. P. (1998). Non-alcoholic steatohepatitis (NASH): a disease of emerging identity and importance. *Journal of Hepatology*.

[28] Hotamisligil G. S. (2006). Inflammation and metabolic disorders. *Nature*.

[29] Cui X., Qian D. W., Jiang S., Shang E. X., Zhu Z. H., Duan J. A. (2018). Scutellariae radix and coptidis rhizoma improve glucose and lipid metabolism in T2DM rats via regulation of the metabolic profiling and MAPK/PI3K/akt signaling pathway. *International Journal of Molecular Sciences*.

[30] Mendez-Frausto G., Romero-Aguilera G., Sanchez-Gutierrez R. (2021). B regulatory cells associated with changes in biochemical and inflammatory parameters in normal-glycemic individuals, pre-diabetes and T2DM patients. *Diabetes Research and Clinical Practice*.

[31] Wan J., Benkdane M., Teixeira-Clerc F. (2014). M2 Kupffer cells promote M1 Kupffer cell apoptosis: a protective mechanism against alcoholic and nonalcoholic fatty liver disease. *Hepatology*.

[32] Kim M. B., Lee Y., Bae M. (2021). Sugar kelp (Saccharina latissima) inhibits hepatic inflammation and fibrosis in a mouse model of diet-induced nonalcoholic steatohepatitis. *The Journal of Nutritional Biochemistry*.

[33] Firmal P., Shah V. K., Chattopadhyay S. (2020). Insight into TLR4-mediated immunomodulation in normal pregnancy and related disorders. *Frontiers in Immunology*.

[34] Zhou Y., Ma X. Y., Han J. Y. (2021). Metformin regulates inflammation and fibrosis in diabetic kidney disease through TNC/TLR4/NF-*κ*B/miR-155-5p inflammatory loop. *World Journal of Diabetes*.

[35] Guo X., Shi Y., Du P. (2019). HMGB1/TLR4 promotes apoptosis and reduces autophagy of hippocampal neurons in diabetes combined with OSA. *Life Sciences*.

[36] Zhang Z., Schluesener H. J. (2006). Mammalian toll-like receptors: from endogenous ligands to tissue regeneration. *Cellular and Molecular Life Sciences*.

[37] Kawai T., Akira S. Z. (2007). Signaling to NF-*κ*B by toll-like receptors. *Trends in Molecular Medicine*.

[38] Ruland J. (2011). Return to homeostasis: downregulation of NF-*κ*B responses. *Nature Immunology*.

[39] Wang L., Guo J., Zhou J., Wang D., Kang X., Zhou L. (2020). NF-*κ*B maintains the stemness of colon cancer cells by downregulating miR-195-5p/497-5p and upregulating MCM2. *Journal of Experimental & Clinical Cancer Research*.

[40] Tapryal N., Shahabi S., Chakraborty A. (2021). Intrapulmonary administration of purified NEIL2 abrogates NF-*κ*B-mediated inflammation. *Journal of Biological Chemistry*.

[41] Mukherjee S., Karmakar S., Babu S. P. S. (2016). TLR2 and TLR4 mediated host immune responses in major infectious diseases: a review. *Brazilian Journal of Infectious Diseases*.

